The article "Functional Role of mTORC2 versus Integrin-Linked Kinase in Mediating Ser473-Akt Phosphorylation in PTEN-Negative Prostate and Breast Cancer Cell Lines" was retracted in 2018. Reasons: fabricated or falsified data; fabricated or falsified images; an official misconduct investigation; misconduct by an author.

# Functional Role of mTORC2 versus Integrin-Linked Kinase in Mediating Ser473-Akt Phosphorylation in PTEN-Negative Prostate and Breast Cancer Cell Lines

**DOI:** 10.1371/journal.pone.0067149

**Published:** 2013-06-19

**Authors:** Su-Lin Lee, Chih-Chien Chou, Hsiao-Ching Chuang, En-Chi Hsu, Po-Chen Chiu, Samuel K. Kulp, John C. Byrd, Ching-Shih Chen

**Affiliations:** 1 Division of Medicinal Chemistry, College of Pharmacy, The Ohio State University, Columbus, Ohio, United States of America; 2 Division of Hematology, Department of Internal Medicine, The Ohio State University, Columbus, Ohio, United States of America; 3 Institute of Basic Medical Sciences, National Cheng-Kung University, Tainan, Taiwan; Florida International University, United States of America

## Abstract

Although the rictor-mTOR complex (mTORC2) has been shown to act as phosphoinositide-dependent kinase (PDK)2 in many cell types, other kinases have also been implicated in mediating Ser473-Akt phosphorylation. Here, we demonstrated the cell line specificity of integrin-linked kinase (ILK) versus mTORC2 as PDK2 in LNCaP and PC-3 prostate and MDA-MB-468 breast cancer cells, of which the PTEN-negative status allowed the study of Ser473-Akt phosphorylation independent of external stimulation. PC-3 and MDA-MB-468 cells showed upregulated ILK expression relative to LNCaP cells, which expressed a high abundance of mTOR. Exposure to Ku-0063794, a second-generation mTOR inhibitor, decreased Ser473-Akt phosphorylation in LNCaP cells, but not in PC-3 or MDA-MB-468 cells. In contrast, treatment with T315, a novel ILK inhibitor, reduced the phosphorylation of Ser473-Akt in PC-3 and MDA-MB-468 cells without affecting that in LNCaP cells. This cell line specificity was verified by comparing Ser473-Akt phosphorylation status after genetic knockdown of rictor, ILK, and other putative Ser-473-Akt kinases. Genetic knockdown of rictor, but not ILK or the other kinases examined, inhibited Ser473-Akt phosphorylation in LNCaP cells. Conversely, PC-3 and MDA-MB-468 cells were susceptible to the effect of ILK silencing on Ser473-Akt phosphorylation, while knockdown of rictor or any of the other target kinases had no appreciable effect. Co-immunoprecipitation analysis demonstrated the physical interaction between ILK and Akt in PC-3 cells, and T315 blocked ILK-mediated Ser473 phosphorylation of bacterially expressed Akt. ILK also formed complexes with rictor in PC-3 and MDA-MB-468 cells that were disrupted by T315, but such complexes were not observed in LNCaP cells. In the PTEN-functional MDA-MB-231 cell line, both T315 and Ku-0063794 suppressed EGF-induced Ser473-Akt phosphorylation. Inhibition of ILK by T315 or siRNA-mediated knockdown suppressed epithelial-mesenchymal transition in MDA-MB-468 and PC-3 cells. Thus, we hypothesize that ILK might bestow growth advantage and metastatic potential in the course of tumor progression.

The article "Functional Role of mTORC2 versus Integrin-Linked Kinase in Mediating Ser473-Akt Phosphorylation in PTEN-Negative Prostate and Breast Cancer Cell Lines" was retracted in 2018. Reasons: fabricated or falsified data; fabricated or falsified images; an official misconduct investigation; misconduct by an author.

## Introduction

The phosphatidylinositol-3-kinase (PI3K)/Akt signaling axis plays a pivotal role in regulating multiple cellular events including cell growth, survival, metabolism, and motility through the modulation of a plethora of downstream effectors. In response to growth factor or cytokine stimulation, activated PI3K facilitates the production of phosphatidylinositol 3,4,5-trisphosphate, leading to the membrane recruitment and subsequent activating phosphorylation of Akt at Thr308 and Ser473 by phosphoinositide-dependent kinase (PDK)1 and PDK2, respectively. In contrast to the well-characterized PDK1 [1], the molecular identity of PDK2 remains elusive [2]. Although recent evidence has demonstrated that the rictor-mTOR complex (mTORC2) acts as the PDK2 in many types of nonmalignant and tumor cells [3], [4], a number of other kinases have also been implicated in mediating Akt-Ser473 phosphorylation in different cell types [2]. These Ser-473-Akt kinases include integrin-linked kinase (ILK) [5], [6], [7], MAPKAP kinase (MK)2 [8], DNA-dependent kinase (DNA-PK) [9], ataxia telangiectasia mutated (ATM) [10], protein kinase C (PKC)α [11], PKCβII [12], and p21-activated kinase (PAK)1 and PAK2 [13]. Among these putative PDK2s, ILK has received much attention in light of the mechanistic link between aberrant ILK upregulation and tumor progression in many types of human malignancies including those of breast, colon, liver, ovary, pancreas, prostate, stomach, and thyroid [14], [15], [16], [17], [18], [19], [20], [21].

In addition to its ability to mediate the phosphorylation of Akt and glycogen synthase kinase (GSK)3β [5], [6], [7], [22], ILK has been shown to serve as a scaffold protein linking integrins with the actin cytoskeleton [23], and to mediate growth factor/integrin-induced activation of ERKs [24], [25], [26], [27] or p38 [28], [29], [30], [31]. Equally important, ILK exhibits a unique ability to modulate the expression of growth factor receptors, including human epidermal growth factor receptor (HER)2 and epidermal growth factor receptor (EGFR), through the oncoprotein Y box-binding protein (YB)-1 [32], providing a link with growth factor receptor signaling. However, despite recent advances in understanding the tumor-promoting function of ILK, an issue that remains in dispute is whether ILK has kinase activity [33], [34]. For example, genetic studies in various nonmalignant cell types, including chondrocytes [35], fibroblasts [36], and keratinocytes [37], and, more recently, in mice [38] indicate that ILK deletion or mutation did not alter Akt or GSK-3β phosphorylation. In contrast, other studies have demonstrated the suppressive effect of targeted ILK excision on Akt-Ser473 phosphorylation in macrophages [22], the heart [39], skeletal muscle [40], and the peripheral nervous system [41]. Moreover, siRNA-mediated silencing of ILK in MDA-MB-231, PC-3, and other cell lines examined resulted in inhibition of Ser473-Akt phosphorylation and induction of apoptosis [42], [43], and the small-molecule inhibitors of ILK, QLT0267 [21], [32], [42], [43], [44], [45], [46], [47], [48], [49], [50] and T315 [compound **22** in ref. [51]], exhibited *in vitro* and/or *in vivo* antitumor efficacy in various types of cancer cells, in part, by targeting Akt activation. Equally important, recent evidence indicates that ILK forms complexes with rictor in PC-3 and MDA-MB-231 cells, and that this complex formation might play a role in regulating the ability of ILK to promote Akt phosphorylation and cancer cell survival and aggressive phenotype [42], [52].

The article "Functional Role of mTORC2 versus Integrin-Linked Kinase in Mediating Ser473-Akt Phosphorylation in PTEN-Negative Prostate and Breast Cancer Cell Lines" was retracted in 2018. Reasons: fabricated or falsified data; fabricated or falsified images; an official misconduct investigation; misconduct by an author.

Together, these seemingly contradictory data raise a possibility that ILK is responsible for Ser473-Akt phosphorylation in a cell line- and/or cellular context-specific manner. In this study, we used small-molecule inhibitors and genetic knockdown to examine the role of mTORC2 versus ILK as the PDK2 in PTEN-negative LNCaP and PC-3 prostate and MDA-MB-468 breast cancer cell lines. As Akt phosphorylation is constitutively upregulated in these cell lines, they provided a suitable model to study the regulation of Ser473-Akt phosphorylation independent of growth factor or other external stimuli. Evidence indicates that, while mTORC2 acts as the PDK2 in LNCaP cells, ILK plays a major role in facilitating Ser473-Akt phosphorylation in PC-3 and MDA-MB-468 cells. In addition, we obtained evidence that ILK formed complexes with rictor in PC-3 and MDA-MB-468, but not in LNCaP cells, and that both mTORC2 and ILK might play a role in mediating epidermal growth factor (EGF)-induced Ser473-Akt phosphorylation in PTEN-positive MDA-MB-231 cells. Together, these data indicate the complexity in the cellular regulation of Akt activation in different cell lines.

## Materials and Methods

### Cell culture and reagents

LNCaP and PC-3 prostate cancer and MDA-MB-468 breast cancer cells were purchased from the American Type Culture Collection (ATCC; Manassas, VA), and maintained at 37°C in a humidified incubator with 5% CO_2_ in the following culture media: PC-3 and LNCaP, RPMI 1640; MDA-MB-468, DMEM, all of which contained 10% fetal bovine serum (FBS). T315, an ILK inhibitor recently developed in the authors’ laboratory, was synthesized according to an established procedure [51], and its identity and purity were confirmed by nuclear magnetic resonance spectroscopy (300 MHz), high-resolution mass spectrometry, and elemental analysis. Ku-0063794 and doxycycline were purchased from Chemdea (Ridgewood, NJ) and Sigma-Aldrich (St. Louis, MO), respectively. For *in vitro* studies, stock solutions of T315 and Ku-0063794 were made in DMSO and diluted in culture medium to a final DMSO concentration of 0.1%. Antibodies against various target proteins were purchased from the following commercial sources: Akt, p-^473^S-Akt, p-^308^T-Akt, GSK-3β, p-^9^S-GSK-3β, ILK, p70S6K, p-^389^T-p70S6K, mTOR, rictor, raptor, ATM, DNA-PK, PAK1, PAK2 (Cell Signaling Technology, Inc., Danvers, MA); MK2, PKCα, PKCβII (Santa Cruz Biotechnology, Inc, Santa Cruz, CA); β-actin (MP Biomedicals, Irvine, CA). shRNA for ILK in the pLKO.1 vector was purchased from Sigma-Aldrich. Human ILK full-length cDNA in the pCMV-SPORT6 vector and lentiviral pTRIPz vectors encoding Tet/ON inducible control shRNA or ILK shRNA with a red fluorescent protein (RFP) reporter gene (V2THS_48753) were purchased from Thermo Scientific (Rockford, IL). Control siRNA and siRNAs for ILK, ATM, PAK1, and PAK2 were purchased from Cell Signaling Technology, Inc. The siRNA for MK2, DNA-PK, PKCα, and PKCβII were purchased from Santa Cruz Biotechnology, Inc. The shRNA for rictor in the pLKO.1 vector was purchased from Addgene (Cambridge, MA).

The article "Functional Role of mTORC2 versus Integrin-Linked Kinase in Mediating Ser473-Akt Phosphorylation in PTEN-Negative Prostate and Breast Cancer Cell Lines" was retracted in 2018. Reasons: fabricated or falsified data; fabricated or falsified images; an official misconduct investigation; misconduct by an author.

### Cell viability assay

Effect of test agents on cell viability was assessed by using the 3-(4,5-dimethylthiazol-2-yl)-2,5-diphenyl-2H-tetrazolium bromide (MTT) assay in six replicates. Cells were seeded and incubated in 96-well plates in the respective medium with 10% FBS for 24 h, and then exposed to various concentrations of test agents dissolved in DMSO in 5% FBS-supplemented medium. The medium was removed from each well and replaced by 200 µl of 0.5 mg/ml MTT in 10% FBS-containing medium, and cells were incubated in the CO_2_ incubator at 37°C for 2 h. Supernatants were removed from the wells, and the MTT dye was dissolved in 120 µl/well DMSO. Absorbance at 570 nm was determined on a plate reader. Cell viabilities are expressed as percentages of that in the corresponding vehicle-treated control group.

### Immunoblotting

Cells were seeded in 10-cm plates (1×10^6^ cells/plate), incubated in 10% FBS-supplemented medium (10 mL/plate) for 24 h, and exposed to individual test agents at the indicated concentrations for 24 h. Cells were collected by scraping followed by centrifugation, washed with cold phosphate-buffered saline, and lysed in SDS lysis buffer (1% SDS, 50 mM Tris buffer pH 8.1, 10 mM EDTA) containing cocktails of protease inhibitors (Sigma-Aldrich) and phosphatase inhibitors (0.625 mM glycerophosphate, 1.25 mM NaF, 0.25 mM sodium pyrophosphate, 0.5 mM Na_3_VO_4_). Lysates were sonicated for 10 s to disrupt cellular organelles and genomic DNA, and then centrifuged at 13,200 rpm for 15 min. Equal amounts of proteins, as determined by a colorimetric bicinchoninic acid assay (Pierce, Rockford, IL), were resolved by SDS-PAGE and transferred to nitrocellulose membranes. After blocking with Tris-buffered saline containing 0.1% Tween 20 (TBST) and 5% non-fat milk for 40 min, membranes were probed with primary antibodies at 1∶1000 or 1∶500 dilution in TBST at 4°C for 16 h, followed by goat anti-rabbit or anti-mouse IgG-horseradish peroxidase conjugates at 1∶5,000 and 1∶3,000 dilutions, respectively, for 1 h at room temperature. Proteins were visualized by enhanced chemiluminescence.

The article "Functional Role of mTORC2 versus Integrin-Linked Kinase in Mediating Ser473-Akt Phosphorylation in PTEN-Negative Prostate and Breast Cancer Cell Lines" was retracted in 2018. Reasons: fabricated or falsified data; fabricated or falsified images; an official misconduct investigation; misconduct by an author.

### Transfection via nucleofection

Cells (1×10^6^) were harvested by trypsinization, re-suspended in culture medium, centrifuged at 100 rpm for 10 min, and transfected with various siRNA or plasmids using an Amaxa Nucleofection system (Amaxa Biosystems, Gaithersburg, MD) according to the manufacturer’s instructions. Expression of various siRNA or plasmids was confirmed by immunoblotting analysis of the target proteins.

### Lentiviral transfection

To produce infectious lentiviruses encoding ILK shRNA, 293T cells were co-transfected with a lentiviral pTRIPz vector encoding Tet-inducible ILK shRNA together with 2 packaging vectors (pMD2.G and psPAX) using the calcium phosphate transfection protocol. The virus-containing medium was collected 5 days after transfection. To generate MDA-MB-468 stable clones that express inducible ILK shRNA, cells were seeded in 6-well plates (1×10^6^ cells/well) for 24 h, and infected with 1 mL virus-containing medium in the presence of 10 µg/mL polybrene. After 1 h incubation, spin infection was performed by centrifugation of the plates at 2600 rpm for 1.5 h at 25°C followed by overnight incubation. The transfected cells were re-seeded onto T75 flasks with fresh medium containing puromycin (0.3 µg/mL) for selection of stable clones. After 7 days of selection, the stable cell pools were established, and their purities were monitored by RFP expression via fluorescence microscopy. The expression of ILK shRNA was verified by Western blot analysis of lysates from cells incubated in the absence or presence of doxycycline. For ILK knockdown experiments, MDA-MB-468 stable clones with Tet/ON inducible ILK shRNA were treated with doxycycline (2 µg/mL) for 5 days with replacement of medium every 2 days to induce the expression of shRNAs. Successful silencing of ILK in response to doxycycline-induced shRNA expression was verified by Western blot analysis.

The article "Functional Role of mTORC2 versus Integrin-Linked Kinase in Mediating Ser473-Akt Phosphorylation in PTEN-Negative Prostate and Breast Cancer Cell Lines" was retracted in 2018. Reasons: fabricated or falsified data; fabricated or falsified images; an official misconduct investigation; misconduct by an author.

### Co-immunoprecipitation of ILK-Akt and ILK-rictor complexes

PC-3 cells (2×10^6^) were seeded in 15-cm culture dishes in 10% FBS-supplemented RPMI 1640 medium, incubated for 24 h, and then treated with 2.5 μM T315 or DMSO vehicle control in 5% FBS-containing medium for 24 h. Cells were harvested and lysed in lysis buffer (20 mM Tris-HCl pH 7.5, 150 mM NaCl, 10% Triton X-100, 1 mM phenylmethanesulfonyl fluoride (PMSF), and 1mM Na_3_VO_4_) at 4°C for 30 min. Cell lysates were incubated with protein A/G agarose beads (Santa Cruz Biotechnology) to eliminate nonspecific binding, and aliquots containing equal amounts of proteins were directly analyzed for levels of ILK, p-Ser473-Akt, Akt and/or rictor by immunoblotting (input), or incubated overnight with goat anti-Akt or anti-ILK antibody- or IgG-conjugated agarose beads (Santa Cruz Biotechnology) for immunoprecipitation. Agarose beads were washed three times with wash buffer (20 mM Tris-HCl pH 7.5, 150 mM NaCl, 0.5% Triton X-100) and resuspended in SDS sample buffer (100 mM Tris-HCl, pH 6.8, 4% SDS, 5% β-mercaptoethanol, 20% glycerol, and 0.1% bromophenol blue) for immunoblotting analysis using antibodies against the relevant target proteins.

### ILK kinase assay

The effect of T315 on the kinase activity of immunoprecipitated ILK was determined in an *in vitro* kinase assay using bacterially expressed glutathione S-transferase (GST)-tagged Akt (GST-Akt) as substrate. GST-Akt fusion protein was expressed in *Escherichia coli* strain BL21 (DE3; ATCC) by isopropyl-β-D-thiogalactopyranoside (IPTG; Sigma-Aldrich) induction for 3 h at 37°C. Bacterial cells were lysed in STE buffer (10 mM Tris, pH 8.0, 150 mM NaCl, 1 mM EDTA, 5 mM DTT, and 1 mM PMSF) containing 1 mg/ml lysozyme via sonication on ice for 5 min, and centrifuged at 16,000 rpm for 20 min. The supernatant was exposed to glutathione-Sepharose beads (GE Healthcare) with gentle rocking at 4°C for 2 h, and the glutathione beads were then washed three times with ice-cold PBS buffer. The GST-Akt fusion protein was eluted by reduced glutathione in elution buffer (10 mM glutathione, 50 mM Tris-HCl pH 8.0, 5% glycerol) at room temperature for 15 min. For the preparation of immunoprecipitated ILK, PC-3 cells were lysed as described in the previous section, and equivalent amounts of lysates were immunoprecipitated with ILK antibody or rabbit IgG in the presence of protein A/G agarose at 4°C for 12 h. The resulting immunocomplexes were washed three times with lysis buffer, incubated with DMSO vehicle or T315 at indicated concentrations at room temperature for 10 min, and exposed to 2 mg of GST-Akt and 200 mM of ATP in kinase buffer (50 mM HEPES pH 7.0, 10 mM MgCl_2_, 10 mM MnCl_2_, 2 mM NaF, 1 mM Na_3_VO_4_, 2 mM DTT). After 20 min of incubation at 30°C, the reaction was quenched by adding SDS sample buffer, and equal amounts of proteins were subjected to immunoblotting analysis using antibodies against Akt, p-^473^S-Akt, and ILK.

The article "Functional Role of mTORC2 versus Integrin-Linked Kinase in Mediating Ser473-Akt Phosphorylation in PTEN-Negative Prostate and Breast Cancer Cell Lines" was retracted in 2018. Reasons: fabricated or falsified data; fabricated or falsified images; an official misconduct investigation; misconduct by an author.

### Matrix colony formation assay

Cells were cultured in growth factor–depleted three-dimensional Cultrex Basement Membrane Extract (BME) (Trevigen, Gaithersburg, MD), as previously reported [53]. In brief, cell culture dishes (24-well plates) were pre-coated with undiluted phenol red-free BME. PC-3 cells (10^4^ cells per well) were suspended in 200 µl of serum-free medium, and then mixed with 100 µl of cold BME. The cell suspension was added dropwise to each well. After this bottom cell-containing layer was set, serum-free medium containing DMSO or T315 at indicated concentrations was added on top. Medium was changed every three days. After culture for 6 days, cells were fixed with 4% paraformaldehyde for 20 min. Fixation was quenched by three 10-min washes with 0.75% glycine in PBS, and cells were examined microscopically for colony formation.

### Statistical analysis

Quantitative data from *in vitro* experiments are presented as mean ± SD. All experiments were performed using 3–6 replicates/group in at least three independent experiments. Differences between group means were analyzed by ANOVA followed by Dunnett’s post-hoc test for multiple comparisons.

## Results

### Differential susceptibility of different prostate and breast cancer cell lines to the effect of mTORC2 and ILK inhibitors on Ser473-Akt phosphorylation

To shed light onto the contentious issue of the role of mTORC2 versus ILK as PDK2, we examined the effects of the 2^nd^-generation mTORC inhibitor Ku-0063794 [54] versus the ILK inhibitor T315 [51] on cytotoxicity and Ser473-Akt phosphorylation in three PTEN-negative cell lines, i.e., LNCaP, PC-3, and MDA-MB-468. Ku-0063794 was reported to inhibit the kinase activities of mTORC1/2 with IC_50_ values of ∼10 nM, and, at 100 nM, to effectively block Ser473-Akt phosphorylation [54]. T315 inhibited the kinase activity of immunoprecipitated ILK with IC_50_ of 0.6 µM, and showed *in vitro* efficacy in suppressing the phosphorylation of other ILK downstream targets, including GSK3β and myosin light chain, without affecting that of the mTORC2 substrates serum- and glucocorticoid-induced protein kinase-1 and protein kinase Cα [51]. Moreover, T315 exhibited no appreciable inhibition of a series of signaling kinases, including PDK1, Akt, GSK3β, focal adhesion kinase, cKit, and EGFR [51]. A more thorough kinase profiling analysis is currently underway.

The article "Functional Role of mTORC2 versus Integrin-Linked Kinase in Mediating Ser473-Akt Phosphorylation in PTEN-Negative Prostate and Breast Cancer Cell Lines" was retracted in 2018. Reasons: fabricated or falsified data; fabricated or falsified images; an official misconduct investigation; misconduct by an author.

Despite the high potency of Ku-0063794 in inhibiting mTORC1/2 signaling, its cytotoxicity varied to a great extent among the three cell lines examined (Fig. 1A). Among them, LNCaP cells were most susceptible to the suppressive effect of Ku-0063794 on cell viability (IC_50_, 0.4 µM); however, its antitumor activity leveled off at ≥1 µM with a maximum inhibition of 75% of cell viability. This phenomenon might be attributable to the mTOR inhibition-mediated induction of autophagy, which promotes survival in cancer cells [55]. Compared to LNCaP cells, PC-3 and MDA-MB-468 cells were less sensitive to the antiproliferative effect of Ku-0063794. The maximal levels of inhibition attained by the drug were 50% and 30% for PC-3 and MDA-MB-468, respectively, at concentrations ≥2 µM.

**Figure 1:** Effects of mTORC1/2 inhibition on cytotoxicity and Ser-473-Akt phosphorylation in PTEN-negative cancer cell lines. (A) Differential susceptibility of LNCaP, PC-3, and MDA-MB-468 (468) cells to Ku-0063794-mediated suppression of cell viability in 5% FBS-supplemented medium after 24 h of treatment. Cell viability was determined by MTT assays. *Points*, means; *bars*, SD (n = 6). (B) Dose-dependent inhibitory effects of Ku-0063794 on mTOR signaling, as indicated by p70SK phosphorylation, and Akt phosphorylation at Ser-473 versus Thr-308. Representative blots from three independent experiments are shown.

Mechanistic evidence suggests that this differential sensitivity to Ku-0063794-induced cytotoxicity was attributable to differences between the sensitive and resistant cell lines in their Akt phosphorylation status in response to Ku-0063794 exposure. As shown in Fig. 1B, exposure to Ku-0063794, at 200–800 nM, led to a robust, concentration-dependent decrease in the phosphorylation level of p70S6K in all three cell lines, indicative of its effectiveness in inhibiting mTOR signaling. While this mTOR inhibition was associated with the selective repression of Akt phosphorylation at Ser-473 in LNCaP cells, no appreciable changes were noted in PC-3 or MDA-MB-468 cells, which refutes the link between mTOR signaling and Akt phosphorylation status in these two cell lines.

In contrast, T315 was effective in suppressing the viability of all three cell lines with IC_50_ values in the range of 1.5–2 µM (MDA-MB-468, 1.5 µM; PC-3 and LNCaP, 2 µM) (Fig. 2A). The ability of T315 to inhibit ILK in these cell lines was evident in the dose-dependent suppression of relevant biomarkers, including the phosphorylation of GSK3β [5], [6], [7], [22] and the expression of the oncogenic factor Y-box binding protein (YB)-1 [32], [51], [56] (Fig. 2B). However, the selective downregulation of Akt phosphorylation at Ser-473 by T315 was observed in PC-3 and MDA-MB-468 cells, but not in LNCaP cells (Fig. 2B). These data suggest that mTORC2 and ILK might play mutually exclusive roles in mediating the phosphorylation of Ser473-Akt in these cell lines. This premise was supported by the inability of T315 to enhance Ku-0063794-mediated suppression of Ser473-Akt phosphorylation in LNCaP cells relative to Ku-0063794 alone (Fig. 1B), and vice versa in PC-3 cells (Fig. 2C versus 2B).

The article "Functional Role of mTORC2 versus Integrin-Linked Kinase in Mediating Ser473-Akt Phosphorylation in PTEN-Negative Prostate and Breast Cancer Cell Lines" was retracted in 2018. Reasons: fabricated or falsified data; fabricated or falsified images; an official misconduct investigation; misconduct by an author.

**Figure 2:** Evidence that ILK acts as a Ser-473-Akt kinase in PC-3 and MDA-MB-468 cells. (A) Dose-dependent effect of T315 on the viability of LNCaP, PC-3, and MDA-MB-468 (468) cells in 5% FBS-supplemented medium after 24 h of treatment. Cell viability was determined by MTT assays. *Points*, means; *bars*, SD (n = 6). (B) Dose-dependent effects of T315 on the phosphorylation of Akt at Ser473 versus Thr308 and GSK3β. Suppression of GSK3β phosphorylation served as a marker for T315-mediated ILK inhibition. (C) Left panel, co-treatment with 3 µM T315 did not enhance the ability of Ku-0063793 to inhibit Ser473-Akt phosphorylation in LNCaP cells. Right panel, co-treatment with 0.8 µM Ku-0063793 did not enhance the ability of T315 to inhibit Ser473-Akt phosphorylation in PC-3 cells. Cells were exposed to test agents at the indicated concentrations for 24 h in 5% FBS-supplemented medium. (D) Left, representative Western blot of the phosphorylation and/or expression levels of Akt, ILK, and the components of mTORC complexes mTOR, raptor, and rictor in PC-3, LNCaP, and MDA-MB-468 (468) cancer cell lines. Right, relative expression levels of p-Ser-473- and p-Thr-308-Akt, Akt, ILK, mTOR, raptor, and rictor in PC-3 and MDA-MB-468 cells relative to those in LNCaP cells. Amounts of immunoblotted proteins from three independent experiments were quantitated by densitometry and normalized to β-actin. Signals from phosphorylated Akt were first normalized to that of total Akt and then to that of β-actin. The abundance of each protein in PC-3 and MDA-MB-231 cells was expressed as a percentage of that in LNCaP cells. Values, means; bars, S.D. (n = 3). All immunoblots are representative of three independent experiments. *P<0.05, compared to LNCaP cells.

### Differential expression of ILK and mTOR

Pursuant to these findings, we assessed the relative expression levels of ILK versus mTOR, as well as the mTORC components raptor and rictor, in these cell lines. While all three cell lines exhibited upregulated Akt phosphorylation, at both Ser-473 and Thr-308, consistent with their PTEN-negative functional status, ILK and mTOR were differentially expressed among these cell lines (Fig. 2D). ILK expression levels in PC-3 and MDA-MB-468 cells were approximately threefold to fourfold higher than that in LNCaP cells, while the expression of mTOR in PC-3 was about 60% lower than that in LNCaP and MDA-MB-468 cells (*P*<0.05). It is especially noteworthy that PC-3 and LNCaP cells exhibited an inverse expression profile of ILK versus mTOR, i.e., PC-3 cells were high in ILK but low in mTOR expression, while LNCaP cells showed the opposite pattern. With regard to the mTORC components, while raptor was consistently expressed across these cell lines, the expression levels of rictor were lower in LNCaP cells than in PC-3 and MDA-MB-468 cells (*P*<0.05).

The article "Functional Role of mTORC2 versus Integrin-Linked Kinase in Mediating Ser473-Akt Phosphorylation in PTEN-Negative Prostate and Breast Cancer Cell Lines" was retracted in 2018. Reasons: fabricated or falsified data; fabricated or falsified images; an official misconduct investigation; misconduct by an author.

### mTORC2 is responsible for Ser473 Akt phosphorylation in LNCaP cells, while ILK acts as the PDK2 in PC-3 and MDA-MB-468 cells

The cell line-specific roles of mTORC2 and ILK as PDK2 were further verified by genetic knockdown experiments in LNCaP and PC-3 cells. In addition to ILK and the rapamycin-insensitive component of the mTORC2 complex rictor, we also carried out si/shRNA-mediated knockdown of a series of other kinases that have been implicated in mediating Ser473-Akt phosphorylation, including MK2 [8], DNA-PK [57], ATM [10], PKCα [11], PKCβII [12], and PAK1/2 [13], in different cell systems in response to growth factor or other external stimuli.

Western blot analysis indicates the high efficiency of these si/shRNAs in reducing the expression of the respective target proteins in both cell lines (Fig. 3A and 4A). More importantly, the consequent effects of these knockdowns on Ser473-Akt phosphorylation confirmed the cell line specificity of mTORC2 versus ILK in mediating the PDK2 function in LNCaP and PC-3 cells. As shown, only the knockdown of rictor, but not ILK or any of the other targeted kinases, resulted in a reduction in p-Ser473-Akt expression in LNCaP cells (Fig. 3A). Conversely, this downregulation of Ser473-Akt phosphorylation was highly specific for the siRNA-mediated knockdown of ILK in PC-3 cells (Fig. 4A).

**Figure 3:** Evidence that mTORC2 is the Ser-473-Akt kinase in LNCaP cells. (A) Western blot analysis of the effect of si/shRNA-mediated knockdown of ILK, rictor, MK2, DNA-PK, ATM, PKCα, PKCβII, PAK1, or PAK2 on the expression of individual target proteins and the phosphorylation of Akt at Ser473 versus Thr308. (B) Effects of siRNA-mediated ILK knockdown, alone or in combination with Ku-0063794 (0.4 µM, 24 h), on Akt phosphorylation at Ser473 versus Thr308. (C) Dose-dependent effect of ectopic expression of ILK, alone (left panel) or in combination with Ku-0063794 (0.4 µM, 24 h), on the phosphorylation of Ser473-Akt and GSK3β. All immunoblots are representative of three independent experiments.

The article "Functional Role of mTORC2 versus Integrin-Linked Kinase in Mediating Ser473-Akt Phosphorylation in PTEN-Negative Prostate and Breast Cancer Cell Lines" was retracted in 2018. Reasons: fabricated or falsified data; fabricated or falsified images; an official misconduct investigation; misconduct by an author.

**Figure 4:** Evidence that ILK is the Ser473-Akt kinase in PC-3 and MDA-MB-468 cells. (A) Western blot analysis of the effect of si/shRNA-mediated knockdown of ILK, rictor, MK2, DNA-PK, ATM, PKCα, PKCβII, PAK1, or PAK2 on the expression of individual target proteins and the phosphorylation of Akt at Ser473 versus Thr308. (B) Effects of shRNA-mediated rictor knockdown, alone or in combination with T315 (2 µM, 24 h), on Akt phosphorylation at Ser473 versus Thr308. (C) Western blot analysis of the effect of shRNA-mediated repression of ILK (left) or rictor (right) on the phosphorylation of Akt at Ser473 versus Thr308, GSK3β (ILK target) and p70S6K (mTOR target) in MDA-MB-468 cells. For induction of ILK shRNA, cells stably transfected with a lentiviral vector encoding tetracycline-inducible ILK shRNA (TRE-ILKi) were exposed to 2 µg/ml doxycycline for 5 days. All immunoblots are representative of three independent experiments.

In addition to these si/shRNA data, the involvement of ILK in mediating Ser473-Akt phosphorylation in LNCaP cells was refuted by three lines of evidence. First, as we have already shown, LNCaP cells express a low abundance of ILK relative to the other cell lines examined (Fig. 2D). Second, the siRNA-mediated knockdown of ILK alone in LNCaP cells had no appreciable effect on Ser473-Akt phosphorylation, which, however, was markedly reduced by co-treatment with Ku-0063794 (0.4 µM) (Fig. 3B), consistent with the effect observed after combination treatment with T315 and Ku0063794 (Fig. 2C). Third, ectopic expression of ILK, as evidenced by dose-dependent elevation in GSK3β phosphorylation, had a modest effect on Ser473-Akt phosphorylation in LNCaP cells, but could not rescue cells from Ku-0063794-mediated suppression of Akt phosphorylation (Fig. 3C). Similarly, in PC-3 cells, phosphorylation of Ser473-Akt was unaffected by shRNA-mediated knockdown of rictor, but was inhibited by co-treatment with T315 (Fig. 4B), thereby ruling out the involvement of mTORC2 as PDK2 in this cell line.

Although we employed a similar approach to interrogate the role of ILK in mediating the phosphorylation of Ser473-Akt in MDA-MB-468 cells, this cell line was refractory to siRNA-mediated knockdown of ILK after introduction of the siRNA via nucleofection. Therefore, we generated a stable clone that expressed ILK shRNA from a TRE (tetracycline response element) promoter by transfecting cells with a lentiviral Tet-inducible ILK-shRNA vector. As shown, doxycycline induced the expression of ILK shRNA, as indicated by reduced ILK expression and GSK3β phosphorylation, and downregulated Ser473-specific phosphorylation of Akt (Fig. 4C, left panel). In contrast, silencing of rictor, as indicated by loss of rictor expression and reduced p70S6K phosphorylation, had no effect on the p-Ser473-Akt level (right panel).

The article "Functional Role of mTORC2 versus Integrin-Linked Kinase in Mediating Ser473-Akt Phosphorylation in PTEN-Negative Prostate and Breast Cancer Cell Lines" was retracted in 2018. Reasons: fabricated or falsified data; fabricated or falsified images; an official misconduct investigation; misconduct by an author.

### Evidence that ILK binds and phosphorylates Akt in PC-3 cells

We obtained two lines of evidence that Akt is targeted by ILK for phosphorylation in PC-3 cells. First, the physical interaction between these two kinases was verified by co-immunoprecipitation. Lysates of PC-3 cells that had been treated for 24 h with either T315 or vehicle were analyzed directly for levels of ILK, phospho-Ser473-Akt, and Akt by immunoblotting (input), or were subjected to immunoprecipitation with anti-Akt antibodies or IgG. The levels of ILK, phospho-Ser473-Akt, and Akt in the resulting immunocomplexes were then analyzed by immunoblotting, which showed that ILK recognized and bound Akt, and T315 was able to attenuate the interaction of ILK with Akt. Second, we demonstrated the ability of ILK to directly phosphorylate Akt at Ser-473. Specifically, the kinase activity of ILK was assayed using ILK immunoprecipitated from PC-3 cells and bacterially expressed, GST-tagged Akt as substrate. As shown in Fig. 5B, ILK phosphorylated Akt at Ser-473. Equally important, this ILK-mediated phosphorylation of Ser473-Akt was dose-dependently inhibited by T315 (*P*<0.05).

**Figure 5:** Evidence that ILK binds and phosphorylates Akt in PC-3 cells. (A) Co-immunoprecipitation analysis reveals the association of ILK with Akt in PC-3 cells, which can be attenuated by T315. PC-3 cells were treated with 2.5 µM T315 or DMSO control for 24 h. Equal amounts of cell lysates were immunoblotted (WB) with antibodies against ILK, p-Ser473-Akt, or Akt (Input; lower panel), or were immunoprecipitated (IP) with anti-Akt antibody and protein A/G agarose followed by immunoblotting with antibodies against ILK, p-Ser473-Akt, or Akt (upper panel). (B) Effect of T315 on the kinase activity of ILK. Equal amounts of immunocomplexes obtained by immunoprecipitation of ILK from PC-3 cell lysates were incubated with bacterially expressed GST-Akt and 200 mM of ATP in the presence of DMSO or T315 at indicated concentrations for 20 min, and were then subjected to Western blotting with antibodies against p-Ser-473-Akt, Akt, or ILK. The immunoprecipitation procedure using IgG was performed as control. Left panel, Western blot analysis of the dose-dependent effect of T315 on the kinase activity of ILK. Right panel, relative expression levels of phosphorylated Ser-473-Akt after normalization to total Akt and subtraction from control (time zero). Amounts of immunoblotted proteins from three independent experiments were quantitated by densitometry. The abundance of phosphorylated Ser-473-Akt in T315-treated cells was expressed as a percentage of that in the DMSO control cells (0 µM). Values, means; bars, S.D. (n = 3). All immunoblots are representative of three independent experiments. *P<0.05, compared to DMSO control (0 µM).

The article "Functional Role of mTORC2 versus Integrin-Linked Kinase in Mediating Ser473-Akt Phosphorylation in PTEN-Negative Prostate and Breast Cancer Cell Lines" was retracted in 2018. Reasons: fabricated or falsified data; fabricated or falsified images; an official misconduct investigation; misconduct by an author.

### ILK interacts with rictor in PC-3 and MDA-MB-468, but not in LNCaP cells

Recent evidence revealed an interaction between ILK and rictor in MDA-MB-231 and PC-3 cells, which played a pivotal role in regulating the Ser-473-Akt kinase activity of ILK [42], [52]. Pursuant to this finding, we investigated this complex formation in MDA-MB-468, PC-3 and LNCaP cells. Co-immunoprecipitation analysis indicated that ILK formed complexes with rictor in MDA-MB-468 and PC-3 cells, but not in LNCaP cells (Fig. 6). Moreover, in line with the effect noted with QLT0267 [52], T315 reduced the formation of this complex in both cell lines (Fig. 6).

**Figure 6:** ILK interacts with rictor in PC-3 and MDA-MB-468, but not in LNCaP cells. Co-immunoprecipitation analysis reveals that ILK associates with rictor in MDA-MB-468 and PC-3 cells, which can be attenuated by T315. No such association was observed in LNCaP cells. Cells were treated with 2.5 µM T315 or DMSO control for 24 h. Equal amounts of cell lysates were immunoblotted with antibodies against ILK, rictor or β-actin (Input; lower panels), or were immunoprecipitated (IP) with anti-ILK antibody and protein A/G agarose followed by immunoblotting (WB) with antibodies against ILK or rictor (upper panels).

### Putative role of ILK in promoting invasive phenotype in cancer cells

The cell line-specific role of ILK as PDK2 in PC-3 and MDA-MB-468 cells raised a question with regard to its biological function beyond the regulation of Akt signaling in these cells. As ILK is known to promote the aggressive phenotype of cancer cells, in part, by facilitating epithelial-to-mesenchymal transition (EMT) through Snail upregulation [58], we examined the effect of ILK inhibition by genetic knockdown and T315 (2 µM) on the expression of Snail and the EMT markers E-cadherin and vimentin in PC-3 and MDA-MB-468 cells. As shown, both genetic silencing and pharmacological inhibition of ILK suppressed Snail expression and EMT in these two cell lines, as manifested by the concomitant increase in E-cadherin expression and decrease in vimentin expression (Fig. 6A). This is consistent with our earlier finding that T315 blocked the expression of YB-1 in PC-3 cells [51], which plays a pivotal role in facilitating EMT through translational activation of Snail and other EMT-inducing transcriptional factors [59]. Moreover, the suppressive effect of T315 on the invasive phenotype of PC-3 cells was investigated using the basement membrane matrix colony formation assay, which has been used frequently to assess the metastatic capacity of cancer cells [60]. As shown, T315 inhibited the ability of the aggressive PC-3 cells to form colonies in the basement membrane matrix (Fig. 5C). PC-3 cells formed large colonies with stellate morphology, indicative of invasiveness [60], in the control group (DMSO), but T315, at 1 and 2 µM, was effective in blocking this invasive colony formation. Together, these findings suggest a potential functional role of ILK in promoting survival signaling and aggressive phenotype in cancer cells through distinct pathways.

The article "Functional Role of mTORC2 versus Integrin-Linked Kinase in Mediating Ser473-Akt Phosphorylation in PTEN-Negative Prostate and Breast Cancer Cell Lines" was retracted in 2018. Reasons: fabricated or falsified data; fabricated or falsified images; an official misconduct investigation; misconduct by an author.

### Role of ILK versus mTORC2 in mediating epidermal growth factor (EGF)-induced Ser473-Akt phosphorylation in MDA-MB-231 cells

As the results above were generated using PTEN-deficient cell lines, one might raise a question of whether the cell line-specific function of ILK versus mTORC2 as PDK2 was associated with the loss of PTEN function in these cells. To address this issue, we investigated the effects of T315 and Ku-0063794 on EGF-induced Ser473-Akt phosphorylation in the PTEN-functional MDA-MB-231 cells. Earlier studies have demonstrated the key role of ILK in mediating endogenous Ser473-Akt phosphorylation in this cell line [42], [43] as it was susceptible to inhibition by QLT-0267 [42], [43] and T315 [51]. As shown in Fig. 7C, exposure of MDA-MB-231 cells to EGF (150 ng/ml) gave rise to robust increases in the phosphorylation of Akt at both Ser473 and Thr308. Ku-0063793 and T315 effectively reduced the EGF-induced phosphorylation of Ser473-Akt to the basal level, while Thr308-Akt phosphorylation was unaffected by either agent. These data suggest the involvement of both ILK and mTORC2 in facilitating Ser473-Akt phosphorylation in response to EGF in MDA-MB-231 cells, indicating that their PDK2 activity is not dependent upon the lack of PTEN function.

**Figure 7:** Pharmacologic inhibition or genetic silencing of ILK suppresses EMT and invasive phenotype. (A) Inhibition of ILK by si/shRNA-mediated silencing or treatment with T315 reduces the expression of Snail in association with an increase in that of E-cadherin and concomitant reduction in that of vimentin in PC-3 (left panel) and MDA-MB-468 (right panel) cells. Cells were treated with T315 for 24 h. For induction of ILK shRNA, MDA-MB-468 cells stably transfected with a lentiviral vector encoding tetracycline-inducible ILK shRNA (TRE-ILKi) were exposed to 2 µg/ml doxycycline for 5 days. Immunoblots are representative of three independent experiments. (B) Images of invasive colonies after growth of PC-3 cells on basement membrane matrix for 6 days in the presence of DMSO control versus T315 at the indicated concentrations. Bars, 100 μm. (C) Dose-dependent effects of T315 and Ku-0063794 on the EGF-induced phosphorylation of Akt at Ser-473 versus Thr-308 in the PTEN-functional MDA-MB-231 cell line. Cells were co-treated with inhibitor and EGF for 24 h. Representative blots from three independent experiments are shown.

The article "Functional Role of mTORC2 versus Integrin-Linked Kinase in Mediating Ser473-Akt Phosphorylation in PTEN-Negative Prostate and Breast Cancer Cell Lines" was retracted in 2018. Reasons: fabricated or falsified data; fabricated or falsified images; an official misconduct investigation; misconduct by an author.

## Discussion

Although substantial evidence indicates the pivotal role of mTORC2 in mediating Ser473-Akt phosphorylation in different types of nonmalignant and cancer cells, other kinases have also been implicated to function as the Ser473-specific Akt kinase in a cellular context- or cell line-dependent manner. For example, DNA-PK has been shown to act as the Ser473-Akt kinase in the nucleus in response to DNA double-strand breaks in human umbilical vascular endothelial cells [9]. In contrast, in MCF-7 cells, while mTORC2 mediated β1 integrin-induced Ser473-Akt phosphorylation, PAK1/2 was responsible for this phosphorylation in response to other stimuli, including lysophosphatidic acid and platelet-derived growth factor [13]. In this study, we interrogated the role of mTORC2 versus ILK in mediating the phosphorylation of Ser473-Akt in PTEN-negative LNCaP, PC-3, and MDA-MB-468 cells in light of their constitutive activation of Akt. Relative to PTEN-functional cells, these cell lines require no external stimulation to induce Akt activation, which allowed the cell context-independent study of Akt regulation by upstream kinases. Moreover, these cell lines differ with respect to their invasive phenotypes, i.e., non-invasive LNCaP cells versus moderately invasive MDA-MB-468 and highly invasive PC-3 cells. By using pharmacological inhibitors and genetic knockdown, we demonstrated the cell line specificity of mTORC2 and ILK in facilitating Ser473-Akt phosphorylation in these cell lines. Moreover, reminiscent of that reported in MDA-MB-231 cells [42], [52], our data indicate the interaction of ILK with rictor in MDA-MB-468 and PC-3 cells, which, however, was not found in LNCaP cells. This discrepancy might reflect a low abundance of rictor in LNCaP cells (Fig. 2D), which could underlie the inability of ILK to regulate Ser-473-Akt phosphorylation in these cells. Nevertheless, despite lack of Akt inactivation, LNCaP cells were still susceptible to T315-mediated inhibition of cell proliferation, in part, due to the drug’s ability to target other downstream signaling effectors of ILK, including the dephosphorylating activation of GSK3β and reduction of the expression of the oncoprotein YB-1 (Fig. 2B). GSK3β activation in response to various cellular stresses has been shown to induce apoptosis by facilitating the proteasomal degradation of key signaling proteins governing survival and cell cycle progression, including β-catenin and cyclin D1 [61]. In addition, GSK3β has been reported to function as a repressor of androgen receptor-mediated transactivation and cell growth in LNCaP cells [62]. Moreover, the role of YB-1 in regulating cancer cell growth survival is well recognized as siRNA-mediated depletion of YB-1 has been shown to induce apoptosis in many cancer cell lines [63]. Thus, the effects on these two signaling effectors might underlie the high *in vitro* efficacy of T315 in suppressing the proliferation of LNCaP cells.

The article "Functional Role of mTORC2 versus Integrin-Linked Kinase in Mediating Ser473-Akt Phosphorylation in PTEN-Negative Prostate and Breast Cancer Cell Lines" was retracted in 2018. Reasons: fabricated or falsified data; fabricated or falsified images; an official misconduct investigation; misconduct by an author.

Although this investigation was conducted in a limited number of PTEN-negative cell lines, the proposed function of ILK in promoting cancer cell aggressiveness is consistent with recent reports that link upregulation of ILK expression with tumor metastasis and progression in prostate cancer, breast cancer, and many other types of human malignancies [14], [15], [16], [17], [18], [19], [20], [21]. Moreover, ILK upregulation has been reported to be a cellular response to various stimuli in the tumor environment leading to activation of Akt signaling in cancer cells, including human leukemic cells co-cultured with bone marrow-derived stromal cells [27], hepatocellular or renal carcinoma cells exposed to hypoxia [64], ovarian cancer cells treated with peritoneal tumor fluids [17], and MDA-MB-231 cells undergoing transforming growth factor β-1-induced EMT [52]. Together, these findings raise a possibility that in the course of tumor progression, cancer cells upregulate the expression of ILK in response to microenvironmental stimuli, such as hypoxia and inflammatory cytokines, to gain growth advantage and metastatic capacity mediated through various downstream signaling effectors, including Akt, GSK3β, and YB-1 [23], [32], [65], [66]. For example, as GSK3β inhibition upregulates Snail, a transcriptional repressor of E-cadherin, ILK activation leads to the transition of cancer cells from an epithelial to mesenchymal phenotype [58]. Moreover, ILK activates the expression of YB-1, which facilitates EMT through the translational activation of Snail and other EMT-inducing transcription factors [59]. This premise is supported by the finding that genetic knockdown or pharmacological inhibition of ILK could inhibit EMT, in part, through the suppression of Snail expression in PC-3 and MDA-MB-468 cells.

In conclusion, the present study demonstrates that ILK mediates Ser473-Akt phosphorylation in PTEN-negative PC-3 and MDA-MB-468 cells. As ILK plays an intricate role in diverse cellular functions associated with survival, proliferation, motility, EMT, and angiogenesis [65], [66], [67], the adoption of ILK as PDK2 might bestow growth advantage and metastatic potential on cancer cells in the course of tumor progression. From a therapeutic perspective, ILK represents an important target for the treatment of metastatic cancer, of which the proof-of-concept is being investigated by using the ILK inhibitor T315 in different tumor models.
